The article "Lung Cancer Classification and Prediction Using Machine Learning and Image Processing" was retracted in 2024. Reasons: signs of a paper mill; compromised peer review; unreliable results or conclusions.

# Lung Cancer Classification and Prediction Using Machine Learning and Image Processing

**DOI:** 10.1155/2022/1755460

**Published:** 2022-08-22

**Authors:** Sharmila Nageswaran, G. Arunkumar, Anil Kumar Bisht, Shivlal Mewada, J. N. V. R. Swarup Kumar, Malik Jawarneh, Evans Asenso

**Affiliations:** ^1^Department of Sensor and Biomedical Technology, School of Electronics Engineering, Vellore Institute of Technology, Tamil Nadu, India; ^2^Department of Computer Science and Engineering, Madanapalle Institute of Technology & Science, Madanapalle, Andhra Pradesh, India; ^3^Department of CS&IT, MJP Rohilkhand University, Bareilly, U. P., India; ^4^Department of Computer Science, Govt. College, Makdone (Vikram University), Ujjain, India; ^5^Department of CSE, SR Gudlavalleru Engineering College, Gudlavalleru, India; ^6^Faculty of Computing Sciences, Gulf College, Oman; ^7^Department of Agricultural Engineering, University of Ghana, Ghana

## Abstract

Lung cancer is a potentially lethal illness. Cancer detection continues to be a challenge for medical professionals. The true cause of cancer and its complete treatment have still not been discovered. Cancer that is caught early enough can be treated. Image processing methods such as noise reduction, feature extraction, identification of damaged regions, and maybe a comparison with data on the medical history of lung cancer are used to locate portions of the lung that have been impacted by cancer. This research shows an accurate classification and prediction of lung cancer using technology that is enabled by machine learning and image processing. To begin, photos need to be gathered. In the experimental investigation, 83 CT scans from 70 distinct patients were utilized as the dataset. The geometric mean filter is used during picture preprocessing. As a consequence, image quality is enhanced. The *K*-means technique is then used to segment the images. The part of the image may be found using this segmentation. Then, classification methods using machine learning are used. For the classification, ANN, KNN, and RF are some of the machine learning techniques that were used. It is found that the ANN model is producing more accurate results for predicting lung cancer.

## 1. Introduction

One of the most lethal types of the disease, lung cancer, is responsible for the passing away of about one million people every year. The current state of affairs in the world of medicine makes it absolutely essential to perform lung nodule identification on chest CT scans. This is due to the fact that lung nodules are becoming increasingly common. As a direct result of this, the deployment of CAD systems is required in order to accomplish the objective of early lung cancer identification [1].

When doing a CT scan, sophisticated X-ray equipment is utilized in order to capture images of the human body from a number of different angles. Following this, the images are fed into a computer, which processes them in such a way as to produce a cross-sectional view of the internal organs and tissues of the body [2].

A CAD approach was trained and assessed in two separate experiments. One research used a computer simulation using ground truth that was generated by computers. In this work, the cardiac-torso (XCAT) digital phantom was used to replicate 300 CT scans. The second research made use of patient-based ground truth using human subjects and implanted spherical nodules of varied sizes (i.e., 3-10 mm in diameter) at random inside the lung area of the simulated pictures. CT images from the LIDC-IDRI dataset were used to create the CAD technique. 888 CT pictures left for processing after CT scans with a wall thickness of more than 2.5 mm were disregarded. In all investigations, a 10-fold cross-validation approach was used to assess network hyperparameterization and generalization. The detection sensitivities were measured in response to the average false positives (FPs) per picture to assess the overall accuracy of the CAD approach. Using the free-receiver response operating characteristic (FROC) curve, the detection accuracy in the patient research was further evaluated in 9 previously published CAD investigations. The mean and standard error between the anticipated value and ground truth were used to measure the localization and diameter estimate accuracies. In all investigations, the average outcomes throughout the 10 cross-validation folds showed that the CAD approach had a high level of detection accuracy. In the patient trial, the corresponding sensitivities were 90.0 percent and 95.4 percent, showing superiority in the FROC curve analysis over many traditional and CNN-based lung nodule CAD approaches. In both investigations, the nodule localization and diameter estimation errors were fewer than 1 mm. The CAD approach that was created was highly efficient in terms of computing [3].

It is likely that intravenous injection of contrast (X-ray dye) may considerably improve the quality of CT imaging, which can reveal a wide variety of organs and tissues. This is one of the potential benefits of contrast injection. In addition, CT scans can reliably detect kidney or gallstones, as well as abnormal fluid buildup or enlarged lymph nodes in the abdominal region or pelvis. This is in addition to the capacity to detect gallstones and kidney stones. Because the CT scan is unable to provide a precise diagnosis of certain organs, such as the stomach, it can, however, be used to reveal abnormalities in the soft tissues that are positioned nearby, offering an indirect diagnosis of these organs [4, 5].

If lung cancer is detected at an early stage, the American Cancer Society estimates that a patient has a 47 percent chance of surviving the disease. It is quite unlikely that X-ray pictures may accidentally reveal lung cancer in its earlier stages [6]. It is famously difficult to detect lesions that are round and have a diameter of 510 millimeters or less. A CT scan of a patient diagnosed with lung cancer is shown in Figure 1.

The processing of images is an essential activity for a diverse variety of business sectors. It is utilized in X-ray imaging of the lungs in order to find regions that contain cancerous growths. In order to detect areas of the lung that have been affected by cancer, image processing techniques such as noise reduction, feature extraction, identification of damaged regions, and maybe a comparison with data on the medical history of lung cancer are utilized. The majority of the time, digital image processing makes use of a diverse set of methods to merge a number of distinct aspects of a picture into a single coherent entity. This research takes an innovative technique in order to zero down on a particular aspect of the overall lung image. The split region may be seen in a variety of ways, including from different viewpoints and when illuminated in different ways. When utilizing this method, one of the key benefits is the ability to differentiate between portions of a picture that have been impacted by cancer and sections that have not been affected by cancer by comparing the intensity of the two sets of photos [6, 7].

As a result of the fact that the majority of patients are diagnosed at a more advanced stage, lung cancer is the primary cause of death resulting from cancer. There is currently no chance of a successful treatment being developed. Lung cancer is consistently ranked as one of the most lethal forms of the disease, regardless of whether a country is industrialized or developing. The incidence of lung cancer in developing countries is on the rise as a result of a longer life expectancy, more urbanization, and the adoption of Western lifestyles. The early detection of cancer and the survival of people with the disease are both essential to the control of lung disease [8, 9].

The literature survey section contains a review of various techniques for the classification and detection of cancer using image processing and classification. The methodology section presents accurate classification and prediction of lung cancer using machine learning and image processing-enabled technology. First, images are acquired. Then, images are preprocessed using the geometric mean filter. This results in improving image quality. Then, images are segmented using the *K*-means algorithm. This segmentation helps in the identification of the region of interest. Then, machine learning classification techniques are applied. The result section contains details related to the dataset and results achieved by various techniques.

To reduce the amount of data that has to be broken down, this study illustrates a method to separate the lung tissue from a chest CT. We will likely have a fully automated computation for cutting the lung tissue into sections and for separating the two sides of the lung as well. The threshold shown in the image separates fat from low-thickness tissue (the lungs). Cleaning is done to get rid of the commotion, air, and flight routes. Finally, a combination of morphological operations is used to tame the unexpected limit. The database used for the evaluation was obtained from a book that instructs radiologists. The current analysis shows that the linked division computation attempts to handle a wide range of different circumstances. The portioned lungs' textural accents were taken off, and it was provided. The neurological system is used to differentiate between the various lung diseases [10].

### 1.1. Literature Survey

Palani and Venkatalakshmi [11] have given predictive modeling of lung cancer illness by continuous monitoring. They did this by using fuzzy cluster-linked augmentation with a categorization. The fuzzy clustering approach is essential to the production of accurate picture segmentation. We instead utilized the fuzzy *C*-means clustering approach in order to accomplish our goal of further disentangling the characteristics of the transitional area from those of the lung cancer image. In this particular investigation, the Otsu thresholding method was applied in order to distinguish the transition area from the lung cancer representation. In addition to this, the right edge picture is utilized in conjunction with the morphological, thinning procedure in order to improve the presentation of the segmentation. The current Association Rule Mining (ARM), the conventional decision tree (DT), and the CNN are combined with a novel incremental classification technique in order to accomplish classification in an incremental fashion. In order to carry out the operations, standard images from the database were utilized, as well as the most recent data on the patient's health collected from IoT devices that were attached to the patient. The culmination of the research indicates that the predictive modeling system has become more accurate.

Deep residual learning was utilized by Bhatia et al. in order to develop a method for determining whether or not a CT picture contains lung cancer. The researchers have devised a preprocessing pipeline by making use of the UNet and ResNet models. This pipeline is intended to highlight and extract features from sections of the lung that are cancerous. An ensemble of XGBoost and random forest classifiers is used to gather predictions about the likelihood that a CT scan is malignant. The results of each classifier's predictions are then pooled, and the final result is used to determine the likelihood that a CT scan is malignant. The LIDC-IRDI has an accuracy that is 84 percent higher than that of typical techniques [12].

Joon et al. [13] segmented lung cancer using an active spline model as their method of analysis. With X-ray photos, through the use of this technique, X-ray images of the lung have been obtained. To begin, it is recommended that a median filter be used for noise detection while the preprocessing stage is being carried out. During the phase devoted to segmentation, further *K*-means and fuzzy *C*-means clustering are utilized for the purpose of feature capture. In this research, the ultimate feature retrieval outcome is reached after the X-ray picture has been segmented. The recommended model was developed by the application of the SVM approach for classification. In order to simulate the findings of the cancer detection system, MATLAB is utilized. The purpose of this study was to detect and categorize lung cancer by making use of images that were both normal and malignant.

Nithila and Kumar [14] have developed an active contouring model, and this model has been deployed. An application of a variation level set function was used for the segmentation of the lungs. It is essential to properly segment the parenchyma in order to arrive at an appropriate diagnosis of lung illness. CT, which stands for computerized tomography, was the first imaging modality to make use of image analysis in this manner. A significant advancement in CT lung image segmentation has been made by the development of the SBGF-new SPF function, which stands for selective binary and Gaussian filtering-new signed pressure force. By taking this strategy, external lung limitations have been identified, and inefficient expansion at the margins has been prevented. Comparisons are being made between the currently under consideration algorithm and four distinct active contour models. The results of the tests demonstrate that the strategy that was provided is reliable and can be computed very quickly [13].

Lakshmanaprabu et al. [15] created OODN (Optimal Deep Neural Network) by lowering the number of characteristics in lung CT scans and comparing it to other classification algorithms. This allowed them to design a more accurate method. The adoption of an automated classification method for lung cancer has cut down on the amount of time needed for human labeling and removed the possibility of mistakes being made by the individual doing the labeling. According to the findings of the researchers, the performance of the machine learning algorithms in terms of accuracy and precision in the detection of normal and abnormal lung photos has significantly increased. According to the findings, the research was successful in classifying lung pictures with a peer specificity of 94.56 percent, a level of accuracy of 96.2 percent, and a level of sensitivity of 94.2 percent. It has been shown that it is feasible to increase the performance of cancer detection in CAT scans [14]. The research has shown that this is the case.

Talukdar and Sarma have placed a strong emphasis on the use of image processing methods for the diagnosis of lung cancer (2018). Deep learning methodologies are being applied to the study of lung cancer. The most prevalent kind of cancer, lung cancer, is taking the lives of an alarmingly high number of individuals. The likelihood of an individual acquiring lung cancer was evaluated with a computed tomography (CT) scan. The growth of precancerous tissue is referred to as “nodules,” and their presence is utilized as a general indication of cancer. Educated radiologists are able to detect nodules and often predict their relationship with cancer. However, these radiologists are also capable of producing false positive and false negative findings. Because the patient is under continual stress, a tremendous quantity of data is evaluated, and a decision that is suitable for the patient is made in a timely manner. As a consequence of this, developing a computer-aided detection system that is capable of rapidly detecting features based on the input of radiologists is most likely to be the answer [15].

Yu et al. have obtained histopathology whole-slide slides of lung cancer and squamous cell carcinoma that have been stained with hematoxylin and eosin (2016). Patients' photographs were taken from TCGA (The Cancer Genome Atlas) and the Stanford TMA (Tissue Microarray Database), plus an additional 294 photos. Even when conducted with the greatest of intentions, an assessment of human pathology cannot properly predict the patient's prognosis. A total of 9,879 quantitative elements of an image were retrieved, and machine learning algorithms were used to select the most important aspects and differentiate between patients who survived for a short period of time and those who survived for a long period of time after being diagnosed with stage I adenocarcinoma or squamous cell carcinoma. The researchers used the TMA cohort to validate the survival rate of the recommended framework (P0.036 for tumor type). According to the findings of this study, the characteristics that are created automatically may be able to forecast the prognosis of a lung cancer patient and, as a consequence, may help in the development of personalized medication. The methodologies that were outlined can be utilized in the analysis of histopathology images of various organs [16].

Pol Cirueda and his colleagues used an aggregation of textures that kept the spatial covariances across features consistent. Mixing the local responses of texture operator pairs is done using traditional aggregation functions like the average; nonetheless, doing so is a vital step in avoiding the problems of traditional aggregation. Pretreatment computed tomography (CT) scans were utilized in order to assist in the prediction of NSCLC nodule recurrence prior to the administration of medication. After that, the recommended methods were put to use in order to compute the kind of NSCLC nodule recurrence according to the manifold regularized sparse classifier. These discoveries, which offer up new study possibilities on how to use morphological, tissue traits to evaluate cancer invasion, need to be confirmed and investigated further. However, this will not be possible without more research. When modeling orthogonal information, the author focused on the textural characteristics of nodular tissue and coupled those characteristics with other variables such as the size and shape of the tumor [17].

The creation of a method for the early detection and accurate diagnosis of lung cancer that makes use of CT, PET, and X-ray images by Manasee Kurkure and Anuradha Thakare in 2016 has garnered a significant amount of attention and enthusiasm. The utilization of a genetic algorithm that permits the early identification of lung cancer nodules by diagnostics allows for the optimization of the findings to be accomplished. It was necessary to employ both Naive Bayes and a genetic algorithm in order to properly and swiftly classify the various stages of cancer images. This was done in order to circumvent the intricacy of the generation process. The categorization has an accuracy rate of up to eighty percent [18].

Sangamithraa and Govindaraju [19] have used a preprocessing strategy in order to eliminate the unwanted unaffected by the use of median and Wiener filters. This was done in order to improve the quality of the data. The *K*-means method is used to do the segmentation of the CT images. EK-mean clustering is the method that is used to achieve clustering. To extract contrast, homogeneity, area, corelation, and entropy features from images, fuzzy EK-mean segmentation is utilized. A back propagation neural network is utilized in order to accomplish the classification [20].

According to Ashwini Kumar Saini et al. (2016), a summary of the types of noise that might cause lung cancer and the strategies for removing them has been provided. Due to the fact that lung cancer is considered to be one of the most life-threatening kinds of cancer, it is essential that it be detected in its earlier stages. If the cancer has a high incidence and mortality rate, this is another indication that it is a particularly dangerous form of the disease. The quality of the digital dental X-ray image analysis must be significantly improved for the study to be successful. A pathology diagnosis in a clinic continues to be the gold standard for detecting lung cancer, despite the fact that one of the primary focuses of research right now is on finding ways to reduce the amount of image noise. X-rays of the chest, cytological examinations of sputum samples, optical fiber investigations of the bronchial airways, and final CT and MRI scans are the diagnostic tools that are utilized most frequently in the detection of lung malignancies (MRI). Despite the availability of screening methods like CT and MRI that are more sensitive and accurate in many parts of the world, chest radiography continues to be the primary and most prevalent kind of surgical treatment. It is routine practice to test for lung cancer in its early stages using chest X-rays and CT scans; however, there are problems associated with the scans' weak sensitivities and specificities [19].

Neural ensemble-based detection is the name given to the automated method of illness diagnosis that was suggested in Kureshi et al.'s research [21] (NED). The approach that was suggested utilized feature extraction, classification, and diagnosis as its three main components. In this experiment, the X-ray chest films that were taken at Bayi Hospital were utilized. This method is recommended because it has a high identification rate for needle biopsies in addition to a decreased number of false negative identifications. As a result, the accuracy is improved automatically, and lives are saved [22].

Kulkarni and Panditrao [23] have created a novel algorithm for early-stage cancer identification that is more accurate than previous methods. The program makes use of a technology that processes images. The amount of time that passes is one of the factors that is considered while looking for anomalies in the target photographs. The position of the tumor can be seen quite clearly in the original photo. In order to get improved outcomes, the techniques of watershed segmentation and Gabor filtering are utilized at the preprocessing stage. The extracted interest zone produces three phases that are helpful in recognizing the various stages of lung cancer: eccentricity, area, and perimeter. These phases may be found in the extracted interest zone. It has been revealed that the tumors come in a variety of dimensions. The proposed method is capable of providing precise measurements of the size of the tumor at an early stage [21].

Westaway et al. [24] used a radiomic approach to identify three-dimensional properties from photos of lung cancer in order to provide prediction information. As is well known, classifiers are devised to estimate the length of time an organism will be able to continue existing. The Moffitt Cancer Center in Tampa, Florida, served as the location from where these photographs for the experiment's CT scans were obtained. Based on the properties of the pictures produced by CT scans, which may suggest phenotypes, human analysis may be able to generate more accurate predictions. When a decision tree was used to make the survival predictions, it was possible to accurately forecast seventy-five percent [23] of the outcomes.

CT (computed tomography) images of lung cancer have been categorized with the use of a lung cancer detection method that makes use of image processing. This method was described by Chaudhary and Singh [25]. Several other approaches, including segmentation, preprocessing, and the extraction of features, have been investigated thus far. The authors have distinguished segmentation, augmentation, and feature extraction, each in its own unique section. In Stages I, II, and III, the cancer is contained inside the chest and manifests as larger, more invasive tumors. By Stage IV, however, cancer has spread to other parts of the body [24], at which point it is said to be in Stage IV.

## 2. Methodology

This section shows an accurate classification and prediction of lung cancer using technology that is enabled by machine learning and image processing. To begin, photos need to be gathered. After that, a geometric mean filter is used to perform preprocessing on the images. This ultimately leads to an improvement in image quality. After that, the *K*-means method is used to segment the images. The identification of the region of interest is facilitated by this segmentation. After that, categorization strategies based on machine learning are utilized.  Figure 2 illustrates the classification and prediction of lung cancer utilizing technology that enables machine learning and image processing.

The preprocessing of images plays a significant role in the proper classification of photographs of illnesses. CT scans provide images with a broad variety of artefacts, including noise, which may be seen in these scans. These artefacts may be removed by using image filtering methods. A geometric mean filter is applied to the input pictures in an effort to decrease the amount of noise [25].

This is accomplished by using a method known as linear discriminant analysis (LDA), which cuts down on the amount of space required for the initial data matrix. The PCA and LDA are two examples of parallel transformation algorithms. In contrast to the supervised LDA method, the PCA is an unsupervised analysis method. In contrast to principal component analysis (PCA), latent dynamic analysis (LDA) seeks to identify a feature subspace that maximizes the possibility of class restoration. It is possible to avoid overfitting by placing more importance on the class-reparability of the data rather than the processing costs [26].

The method of segmentation is used in the process of medical image processing. The basic role of a picture is to differentiate between components that are beneficial and those that are harmful. As a consequence of this, it separates a picture into distinct pieces based on the degree to which each component is similar to its surrounding components. This effect may be achieved by manipulating the intensity as well as the texture. An area of interest that has been segmented may be utilized as a diagnostic tool to quickly get information that is pertinent to the issue at hand. When it comes to the process of segmenting medical pictures, the technique known as *K*-means clustering is the one that is used most often. During the clustering process, the picture is divided into a number of different groups, also known as clusters, which do not overlap with one another. These clusters are not connected to one another in any way. In this picture, there are a few distinct clusters that can be noticed. Every one of them has its own one-of-a-kind collection of reference points to which each pixel is assigned. To divide the available data into *k* separate groups, the *K*-means clustering algorithm divides the available information based on *k* reference points [27].

Artificial neural networks, also known as ANNs, are used often in the medical industry for the purpose of classifying medical images for the goal of diagnosing illness. In terms of the way it performs its tasks, the ANN is fairly comparable to the human brain. It is feasible to get the knowledge required to make an informed guess about the category that a photograph belongs to by looking at a collection of images that have already been categorized. This may be accomplished by looking at a collection of pictures that have been categorized. A category has already been selected for each of the pictures included in this gallery. An artificial neural network (ANN) is constructed up of artificial neurons, which are programmed to behave in a manner that is analogous to that of their biological counterparts in the human brain. Neurons are able to communicate with one another outside of their bodies through connections. It is possible to assign weights to neurons and edges, and those weights may be changed at any time throughout the process of learning. The standard structure of an artificial neural network has three layers: an input layer, a hidden layer, and an output layer that is in charge of creating the signal. This is the architecture that is used the most often. The most popular topologies for artificial neural networks include an input layer, a hidden layer, and a final layer; however, there are other possible configurations as well. It is conceivable that there is just one hidden layer, that there are several hidden levels, or that there are no hidden layers at all. Each and every one of these options is not completely out of the question. The weights that need to be adjusted until the desired output is reached are tucked away in a layer that is below the active layer [28]. The iterations are closely related to computing efficiency during the training of the ANN model. Precision will suffer by having too few hidden layer neurons, while too many neurons would lengthen training time.

The KNN approach, which is the method that is used in ML the most commonly, makes it easy to learn about the algorithms that are employed in ML. It is a technique of supervised learning that does not need the use of any parameters. The phase that the *k*-training NN goes through is thus significantly quicker than the phase that other classifiers go through. The testing stage, on the other hand, takes longer and uses more memory as it goes on. In order to use *k*-nearest neighbors to categorize new kinds of data points, one needs first to have data that is already organized into many different categories. Because training observations are included in each labeled dataset, the algorithm is able to establish a connection between *x* and *y* in each training dataset (*x*, *y*). The typical practice at this location is delaying the processing in order to locate the KNN function. The contributions of neighbors may be weighted in classification models as well as regression models, which can result in a higher average score for those who live in close proximity to one another in comparison to those who live farther away. As the distance between two neighbors increases, an additional weighting of 1/*d* is applied to each neighbor [29]. Despite producing good precision on the test dataset, KNN is still slower and more expensive to run in terms of both time and memory. To store the whole training dataset for prediction, it needs a lot of memory. Additionally, as Euclidean distance is very reactive to orders of magnitude, features in the dataset with high magnitudes always have a higher weight than those with low magnitudes. Last but not least, we must remember that KNN is not appropriate for large-dimensional datasets.

It is possible to construct predictive models by using the random forest approach, which is used by a lot of people. Only two of the many applications that may be accomplished using RF are regression and classification [30]. It is possible to develop machine learning algorithms that are capable of making predictions with a high degree of accuracy so long as datasets are changed appropriately [31]. This approach is highly user-friendly in comparison to other algorithms, and it has a lot of support from members of the general public. For the purposes of this model, RF is an abbreviation for “random forest,” and true to its moniker, the model creates random forests. With the help of this technique, one may generate an entire grove of decision trees, each of which is trained in a distinct way. This method was used to build the current thicket of trees representing the many possible multiple-choice responses. As a direct consequence of this, they were integrated in order to provide even more accurate projections [22].

## 3. Result Analysis

A dataset of 83 CT images from 70 different patients was used in the experimental study [*x*]. Images are preprocessed using the geometric mean filter. This results in improving image quality. Then, images are segmented using the *K*-means algorithm. This segmentation helps in the identification of the region of interest. Then, machine learning classification techniques are applied.

For performance comparison, three parameters, accuracy, sensitivity, and specificity, are used:

(1) $$\begin{array}{c} \text{Accuracy}=\frac{\text{TP}+\text{TN}}{\text{TP}+\text{TN}+\text{FP}+\text{FN}},\\ \text{Sensitivity}=\frac{\text{TP}}{\text{TP}+\text{FN}},\\ \text{Specificity}=\frac{\text{TN}}{\text{TN}+\text{FP}}, \end{array}$$

where TP is true positive, TN is true negative, FP is false positive, and FN is false negative.

Results of different machine learning predictors are shown in Figures 3–5. The accuracy of ANN is better.

## 4. Conclusion

Lung cancer is one of the deadliest types of the disease, claiming the lives of approximately one million people each year. Given the current state of affairs in medicine, it is critical that lung nodule identification be performed on chest CT scans. As a result, the use of CAD systems is crucial for the early detection of lung cancer. Image processing is a necessary activity that is employed in a wide range of economic domains. It is used in X-ray imaging of the lungs to find areas of the body that have developed malignant growths. Image processing techniques such as noise reduction, feature extraction, identification of damaged regions, and maybe comparison with data on the medical history of lung cancer are used to locate sections of the lung that have been affected by cancer. This study demonstrates accurate lung cancer classification and prediction using technologies enabled by machine learning and image processing. To begin, photographs must be collected. Following that, the images are preprocessed using a geometric mean filter. This eventually leads to an increase in image quality. The *K*-means approach is then used to segment the images. This segmentation makes it easier to identify the region of interest. Following that, machine learning-based categorization algorithms are used. ANN predicts lung cancer with more accuracy. This research will help to increase the accuracy of lung cancer detection systems that use strong classification and prediction techniques. This study brings cutting-edge images based on machine learning techniques for implementation purposes.

## Figures and Tables

**Figure 1:** CT scan image for lung cancer.

**Figure 2:** Classification and prediction of lung cancer using machine learning and image processing-enabled technology.

**Figure 3:** Accuracy of machine learning techniques for lung cancer detection.

**Figure 4:** Sensitivity of machine learning techniques for lung cancer detection.

**Figure 5:** Specificity of machine learning techniques for lung cancer detection.

## Data Availability

The data shall be made available on request.
